RETRACTED

# Fumagillin regulates stemness and malignancies in cancer stem-like cells derived from liver cancer via targeting to MetAP-2

**DOI:** 10.1371/journal.pone.0289024

**Published:** 2023-07-28

**Authors:** Ke Zhang, Jian Hu, Ziyi Zhao

**Affiliations:** 1 The Second People’s Hospital of Yibin, Sichuan, China; 2 TCM Regulating Metabolic Diseases Key Laboratory of Sichuan Province, Hospital of Chengdu University of Traditional Chinese Medicine, Sichuan, China; Teikyo University, School of Medicine, JAPAN

## Abstract

**Background:**

Cancer relapse is associated with the presence of cancer stem-like cells (CSCs), which lead to multidirectional differentiation and unrestricted proliferative replication. Fumagillin, a myocotoxin produced by the saprophytic filamentous fungus Aspergillus fumigatus, has been reported to affect malignant characteristics in hepatocellular cancer cells. However, its exact role in CSCs is still unknown.

**Methods:**

CSCs were enriched by culturing cancer cells in serum-free medium. The effects of fumagillin on malignant cell characteristics and mitochondrial function were measured. The regulatory role of fumagillin on methionine aminopeptidase-2 (MetAP-2) was assessed.

**Results:**

When it was supplemented in medium, fumagillin treatment inhibited sphere formation and the maintenance of stemness of CSCs without disturbing cell growth. Fumagillin also decreased stemness-related markers and the aldehyde dehydrogenase 1 (ALDH1)-positive proportion, which demonstrated that fumagillin decreases stemness in CSCs. It was also found to inhibit malignant traits in CSCs, including cell proliferation, invasion, and tumor formation, and sensitize CSCs to chemoagents, including sorafenib and doxorubicin, by promoting chemoagent-induced apoptosis. Moreover, fumagillin treatment was found to disturb mitochondrial membrane homeostasis, ATP synthesis and mitochondrial transcriptional activity. In addition, we found that fumagillin decreased MetAP-2 protein levels and exerted anti-CSC effects potentially by regulating MetAP-2. We also found that fumagillin treatment activated p53 and its transcriptional activity and thus caused cell cycle blockade. Moreover, fumagillin treatment significantly decreased tumor formation in nude mice.

**Conclusion:**

This work offers evidence for fumagillin as a specific inhibitor of liver cancer CSCs and proposes a novel strategy for cancer therapy.

## Introduction

Liver cancer is one of the most common malignant tumors in the digestive system [1]. Liver cancer stem cells (LCSCs) are a small group of cells with self-renewal and multidirectional differentiation potential in liver cancer tissues [2]. LCSCs not only participate in the occurrence and development of liver cancer but also play an extremely important role in the metastasis, recurrence and chemotherapy resistance of liver cancer. In the conventional treatment of liver cancer, usually only proliferating liver cancer cells are eliminated, while LCSCs still exist and can gradually form new tumors, eventually leading to the recurrence of liver cancer [3]. In addition, LCSCs can also enter the circulatory system, migrate and invade distant organs to generate new tumors and promote the formation of tumor metastasis. At the same time, LCSCs show tolerance to a variety of chemotherapy drugs, which is one of the important reasons for chemotherapy resistance in liver cancer.

RETRACTED

Fumagillin, a metabolite with various biological activities, was first isolated from the fermentation medium of Aspergillus fumigatus [4,5] and was originally used to treat microsporidiosis of bees and fish. In 1990, Ingber et al. [6] found that nikotremycin can inhibit tumor angiogenesis, thus blocking the blood supply around tumors, and achieve cancer treatment by covalently modifying HIS-231 at the active site of metap-2 in vivo to inactivate the enzyme. Furthermore, it can specifically inhibit the growth and proliferation of vascular endothelial cells in an irreversible manner. Interestingly, Hou and colleagues also reported its tumor-inhibiting roles in colorectal cancer by inhibiting angiogenesis, indicating its potential antitumor effects in liver cancer [7].

MetAPs are enzymes that remove n-terminal methionine from peptides and proteins. The roles of Metap-2 appear to include protein cotranslation or posttranslation processing and mynutylation, as well as regulation of protein stability [8], which plays an important role in endothelial cell growth [9]. MetAPs are a class of intracellular proteolytic enzymes that play an important role in posttranscriptional and cotranslational modifications of proteins (nutmeg acylation and acetylation of NH2 terminal). In addition, MetAPs are essential new proteins because they control the hydrolysis of iMet at the N-terminus. Proper removal of iMet is also necessary to expose glycine residues where fatty acids can covalently bind, allowing effective binding to membranes or other proteins. Maintaining MetAP activity throughout evolution may have served an energy cycle purpose, since methionine is the most expensive amino acid to synthesize from an energy efficiency standpoint.

Fumagillin is a Metap-2 inhibitor that blocks the formation of blood vessels [10]. SCID mice injected with colon cancer subcortical cells were treated with fumagillin, which resulted in smaller tumors, fewer lung metastases, and lower levels of MVD-CD105 compared with the control group [11]. Quantitative PCR and western blot results showed reduced expression of the cyclin E2, activated leukocyte cell adhesion molecule (ALCAM), and intercellular adhesion molecule 1 (ICAM-1) genes in the presence of fumagillin. This downregulation of fumagillin may be related to the antiangiogenic effect of fumagillin, which inhibits the growth and metastasis of colorectal cancer by inhibiting angiogenesis, indicating that the antitumor effects of fumagillin might be exerted by downregulating the MetAP-2 protein.

RETRACTED

In this paper, we describe the inhibitory roles of fumagillin on the stemness of CSCs derived from liver cancer cells. Fumagillin inhibits MetAP-2 and acts as a potent inhibitor of CSCs. These results indicate that fumagillin is a promising drug for liver cancer that targets CSCs.

## Material and methods

### Cell culture, sphere formation and treatment

Hepatoma cell lines; including Huh-7 and SK-HEP-1, were bought from American Type Culture Collection (ATCC, Manassas, VA, USA). Cells were maintained in RPMI1640 supplemented with fetal bovine serum (FBS, Lonza, Basel, Switzerland), 100 μg/mL streptomycin and 100 units/mL penicillin at 37°C in a humidified, 5% (v/v) CO_2_ atmosphere. Cells were passaged every three days.

To enrich CSCs, cells were cultured in DMEM/F12 medium without FBS, and supplemented with 100 μg/mL streptomycin and 100 units/mL penicillin, 20 ng/ml human recombinant epidermal growth factor (EGF), 20 ng/ml human recombinant basic fibroblast growth factor (bFGF), and 2% B27 supplement (Invitrogen, USA) and seeded in 6-well cell culture plate with ultra-low attachment surface (BioFLOAT, USA). Medium was half-refreshed every three days.

To evaluate the effects of Fumagillin on cell viability, 1, 2.5, 5, 7.5 and 10 μmol/L of Fumagillin, bought from Sigma-Aldrich (USA) in stock at final concentration of 20 mmol/L, was added for 24-hour incubation. To evaluate the effects of Fumagillin on sphere formation, Fumagillin was added for 24–96 h. To evaluate the effects of Fumagillin in maintenance of stemness, Fumagillin was added into spheres.

### Western blot

Total cell protein lysates were extracted using RIPA buffer (0.5 M Tris–HCl, pH 7.4, 1.5 M NaCl, 2.5% deoxycholic acid, 10% NP-40, 10 mM EDTA) by cultured on ice for 10 min. Protein concentration was measured by performing BCA assay (Sigma-Aldrich, USA). 20 μg of total protein was fractionated using 6–12% gradient SDS-PAGE gel using electrophoresis buffer (0.192 M glycine, 25 mM Tris, 0.1% SDS). Fractionated blots were transferred onto a PVDF membrane (Millipore, USA), which was blocked in TBS-T with 5% non-fat dry milk and incubated overnight with the primary antibodies at dilution of 1:1000 as follows: Oct-4 (cat. No.: ab181557), CD44 (cat. No.:ab243894), Sox2 (cat. No.: ab93689), β-actin (cat. No.: ab8226), cleaved Poly [ADP-ribose] polymerase 1 (PARP1, cat. No.: ab32064), cleaved caspase-3 (cat. No.: ab32042), MetAP-2 (cat. No.: ab134124), p53 (cat. No.: ab26), p21 (cat. No.: ab109520). Then membrane was incubated with secondary HRP-linked antibody at dilution of 1:5000. Detection was done by Abcam OptiBlot ECL Detect Kit (Abcam, USA).

RETRACTED

### CCK-8 assay

CCK-8 (Sigma-Aldrich, USA) assay was used to evaluate cell viability. 1×10^4^ cells/well were seeded in 96-well plate. For each well, 10 μl of CCK-8 solution was directly added into the medium (100 μl per well) and incubation at 37°C for 2 h. Wells containing medium only were considered as blank group. The absorbances (Abs) were measured at 450 nm (n = 3). Cell viability = (Abs of experimental group-Abs of blank group)/(Abs of control group-Abs of blank group) × 100%. All experiments have been repeated for three times.

### RT-qPCR

Total RNA was isolated using TRIZol reagent (Life Technology, USA) and complementary DNA (cDNA) was obtained by performing reverse transcription using Quantitect Reverse Transcription Kit (Qiagen, Germany). Quantitative gene expressions were analyzed using FastStart Universal SYBR Green Master (Roche diagnostics, Germany) on a ABI7500 system (Life Technology). PCR condition was as follows: 10 min at 95°C, followed by 35 cycles of 95°C for 30 s and 60°C for 60 s. β-actin was used as an internal control, and expressing level of target genes were calculated using the ΔCq method. Primers used were as follows: COX1 forward 5’- CGTTGTAGCCCACTTCCACT-3’ and reverse 5’- TGGCGTAGGTTTGGTCTAGG-3’; COX3 forward 5’- CAATTACATGAGCTCATCATAGC -3’ and reverse 5’- CCATGGAATCCAGTAGCCA -3’; ND1 forward 5’- CCTAAAACCCGCCACATCTA-3’ and reverse 5’- GCCTAGGTTGAGGTTGACCA-3’; Cyb forward 5’- ATCACTCGAGACGTAAATTATGGCT -3’ and reverse 5’- TGAACTAGGTCTGTCCCAATGTATG -3’; Ubiquitin forward 5’- ATTTGGGTCGCGGTTCTTG -3’ and reverse 5’- TGCCTTGACATTCTCGATGG -3’; β-actin forward 5’- TGCGTTACACCCTTTCTTGACA -3’ and reverse 5’- GCAAGGACTTCCTGTAACAATG -3’.

### ALDH1 staining

To evaluate ALDH1 proportion, cells were collected and washed with PBS containing 0.5% BSA and suspended in concentration of 1×10^6^ cells/ml in 4% formaldehyde solution. Fixed cells were permeabilized using 0.05% Triton X-100 for 10 min at room temperature, which were further blocked using 1 *μ*g of human IgG (Invitrogen)/105 cells for 15 min at room temperature. FITC-conjugated anti-human ALDH1A1 antibody (Sino Biological, Beijing, China) was incubated with blocked cells at dilution of 1:200 for 30 min at room temperature avoiding from light. Fluorescence was measured with a flow cytometer (BD Biosciences, FACSCanto II, San Jose, CA, USA). Isotype-matched human antibodies (BD Biosciences) were used as controls. All experiments have been repeated for three times.

RETRACTED

### PI staining

Cells were collected and washed using pre-cooled PBS solution for 3 times. Cell pellet was fixed using 1 ml of 75% ethyl alcohol and kept overnight at 4°C. Then cells were washed by PBS for 2 times, and incubated with 100 μl RNase A and 400 μl propidium iodide (PI) (Sigma-Aldrich Chemical Company, St Louis, MO, USA) for 30 min at room temperature avoiding from light. Then cells were analyzed with a flow cytometer (BD Biosciences, FACSCanto II, San Jose, CA, USA). Each experiment was repeated 3 times.

### Transwell assay

Transwell invasion assays were performed as described [12]. Cells were seeded in the upper chambers, and conditioned medium was placed in the lower chambers. 48 or 72 hour later, cells were fixed using 4% paraformaldehyde for 15 min at room temperature, then stained with crystal violet and observed under optical microscope. All experiments were performed in triplicate.

### Tumor formation

To evaluate tumor formation ability, soft agar clonogenic assays were done. Briefly, 2 mL of 0.5% (w/v) Noble agar (Difco) in serum-free medium was layed on a 6-well plate. 4×10^3^ cells were mixed in 2 mL of 0.3% (w/v) Noble agar. Plates were incubated (37°C, 5% CO2) under standard conditions for 10 days before colony number and diameter were quantified microscopically.

### Apoptosis analysis

To evaluate apoptotic rate, cells were collected and washed using pre-cooled PBS solution for 3 times. Cells were stained using Annexin V-FITC apoptosis detection kit (Sigma-Aldrich Chemical Company, St Louis, MO, USA). Briefly, 150 μl binding buffer and 5 μl Annexin-V-FITC were added into each tube and well-mixed by shaking, followed by 15 min incubation in the dark. Next, 150 μl binding buffer and 5 μl PI dye (Sigma-Aldrich Chemical Company, St Louis, MO, USA) were added into tube and well-mixed by shaking. Then, cells were analyzed with a flow cytometer (BD Biosciences, FACSCanto II, San Jose, CA, USA). Each experiment was repeated 3 times.

### ATP synthesis

ATP Bioluminescence Assay Kit HS II (Roche Applied Science) was employed to measure intracellular ATP level. 50 μL of Cell lysate was mixed with 50 μL of luciferase reagent followed by thoroughly mix. Then signal was measured and integrated for 10 s by using a SpectraMax M5 luminometer (Molecular Devices).

### JC-1 staining

JC-1 staining followed by flow cytometry analysis was used to detect mitochondrial membrane potential. JC-1 mitochondrial membrane potential assay kit (cat. no., C2006; Beyotime Institute of Biotechnology) was employed. Briefly, collected cells were stained using JC-1 staining solution for 30 min at 37°C followed by flow cytometry analysis using a flow cytometer (BD Biosciences, FACSCanto II, San Jose, CA, USA) [13].

RETRACTED

### In vivo tumor formation

Animal studies were proved by the Medical Ethics Committee of Sichuan University, West China Hospital (No.20220915002). Animal experiment was performed in compliance with the Practice Guidelines for Laboratory Animals of China. Female BALB/c nude mice were bought from Sichuan Dashuo Experimental Animal Company. All mice were kept in microisolator cages in a pathogen-free animal bio-safety level-2 facility at 22±2°C. During the experiments, health monitoring of mice was performed to ensure their health, including monitoring animals from external sources as well as animals kept in the experimental unit; housing and hygienic monitoring, pathogen detection, diagnostic measures to enable disease control and to maintain the health status of mice. After 1 week, the experiment started. Briefly, 5×10^5^ CSCs pretreated with Fumagillin (Fumagillin group) for 48 h or not (Mock group) were seeded in nude mice (n = 4 for each group). Tumor size was measured every five days from day 10 after tumor plant. On day 30, mice were euthanized and beard tumors were pathologically analyzed.

### GEPIA database assay

Gene expression profiling interactive analysis (GEPIA, http://gepia.cancer-pku.cn/) was used to evaluate the expression level of MetAP-2 in LIHC tissues and its association with overall survival rate.

### Statistical analysis

SPSS version 19.0 was used to analyze the data. All data were expressed as the mean ± SEM. Student’s *t*-test was used in the two-group comparisons, and one-way ANOVA was used for more than two groups. *P* value < 0.05 was considered statistically significant.

## Results

### Fumagillin inhibits sphere formation and promotes loss of stemness in CSCs derived from hepatocellular carcinoma cells

To evaluate the effects of Fumagillin on stemness in hepatocellular carcinoma cells, we enriched CSCs from Huh-7 and SNU-449 cells by culturing all these cells in serum-free medium, and growing spheres were observed on day 1, 4, 7, and 10 (Fure 1A). Spheres were obtained on day 10 and characterized by detecting increasing amount of stemness relative markers, including Oct4, CD44 and Sox2 (Fig 1B). By being culture with 1, 2.5, 5, 7.5 or 10 μmol/L Fumagillin for 24h, cell viability was not obviously affected, which promotes us to employ 10 μmol/L of Fumagillin for further investigation (Fig 1C). Then, 10 μmol/L Fumagillin was added into serum-free medium during the process of sphere formation and obviously inhibited sphere formation, without affecting adherent cell growth (Fig 1D).

RETRACTED

**Fig 1:** Fumagillin affects stemness of CSCs derived from hepatocellular carcinoma cells. A. By being cultured in serum-free medium, sphere formation was observed from day 1 to 10 derived from Huh-7 and SNU-449 cells. B. western blot was performed to detect stemness related factors in Huh-7 spheres, including Oct4, CD44, Sox2. *P<0.05, **P<0,01, vs. Parental cell group. C. CCK-8 assay was performed to detect inhibition rate of Fumagillin to cell viability of Huh-7 or SNU-449 CSCs. D. Huh-7 or SNU-449 cells were seeded and allowed to attach overnight. With the presence of Fumagillin for 24–96 h, cell morphology was observed and after 96-hour incubation, stemness related factors in Huh-7 were detected by western blot. *P<0.05, **P<0.01, vs. Mock group.

To further confirm whether Fumagillin induces loss of stemness in CSCs, Fumagillin was into CSC spheres obtained from day 4, and CSCs spheres were cultured for extra 7 days. As it is shown in Fig 2A, Fumagillin expectedly promoted loss of stemness in spheres, which was further confirmed by detecting stemness relative markers (Fig 2B) We further staining stem surface marker of ALDH1 in Fumagillin treated or untreated cells, and observed that Fumagillin treatment significantly decreased ALDH1 positive proportion in both Huh-7 and SNU-449 CSCs (Fig 2C and 2D).

**Fig 2:** Fumagillin affects ALDH1+ positive proportion. A. Spheres were cultured with different concentration of Fumagillin and mophology was observed. B. western blot was performed to detect stemness related factors. *P<0.05, **P<0.01, vs. Mock group. After Fumagillin treatment, ALDH1 staining was performed and analyzed followed by flow cytometry (C&D). *P<0.05, vs. ALDH1+/Fumagillin- group.

### Fumagillin inhibits tumor malignant biological behaviors and sensitizes CSCs to chemoagent

To evaluate whether Fumagillin affects tumor malignant biological behaviors, we firstly cultured Huh-7 and SNU-449 CSCs with 10 μmol/L Fumagillin for 1–5 days, and resulted in significant decrease in cell viability (Fig 3A). Cell cycle analysis also presented that Fumagillin blocked cell cycle at G1 phase, which indicated that Fumagillin decreased cell viability by inhibiting cell proliferation (Fig 3B). We then evaluate the effects of Fumagillin on invasion and tumor formation. Expectedly, Fumagillin treatment remarkably decreased all these behaviors (Fig 3C and 3D), demonstrating that Fumagillin present critical inhibition on malignant biological behaviors.

RETRACTED

**Fig 3:** Fumagillin affects malignant behaviors in CSCs. A. After Fumagillin treatment, cell viability of Huh-7 or SNU-449 CSCs from day 1–5 was measured by performing CCK-8 assay. *P<0.05, vs. Mock group. B. after being treated with Fumagillin for 48 and 72 h, cell cycle distribution of Huh-7 or SNU-449 CSCs was measured by performing PI staining followed by flow cytometry assay. *P<0.05, vs. Mock group. C. After Fumagillin treatment for 48 h, invasion was measured by performing Transwell assay in Huh-7 or SNU-449 CSCs. *P<0.05, vs. Mock group. E. After being co-cultured with Fumagillin for 12 days in soft agar, tumor formation was measured in Huh-7 or SNU-449 CSCs. *P<0.05, vs. Mock group.

Existence of CSCs was thought to be responsible for chemoresistance and recurrence of liver cancer patients [14]. By considering this, we then exposed CSCs to Fumagillin for 24h followed by chemotreatment using sorafenib [15,16] or doxorubicin [17], which are two fist line chemoagents for hepatocellular carcinoma therapy. As it is shown in Fig 4A, Fumagillin pre-treatment promoted cytotoxicity of these two chemoagents. Moreover, Fumagillin pre-treatment significantly increased apoptotic rate induced by doxorubicin or sorafenib (Fig 4B), and increased cleaved PARP1 and caspase-3 (Fig 4C). These results demonstrate that Fumagillin may overcome chemoresistance caused by existence of CSCs.

**Fig 4:** Fumagillin sensitized CSCs to chemoagents. A. Fumagillin was co-cultured with chemoagents, including Sorafenib or Doxorubicin for 24 h, cell viability was measured by performing CCK-8 assay. *P<0.05, vs. Fumagillin group. B. The effects of Fumagillin on sorafenib or Doxorubicin-induced apoptosis were measured by performing Annexin V-FITC/PI double staining followed by flow cytometry. *P<0.05, vs. Doxorubicin group; #P<0.05, vs. Sorafenib group. C. After treatment, apoptosis-specific protein, including cleaved PARP1 and cleaved caspase-3, were detected by performing western blot. *P<0.05, vs. Doxorubicin group; #P<0.05, vs. Sorafenib group.

### Fumagillin induces mitochondrial dysfunction

It is well-established that the stemness of CSCs is tightly associated with elevated glucose and mitochondrial-dependent metabolic activity in several kinds of cancers [18,19]. Notably, Fumagillin was reported to dramatically decreased mitochondrial ATP synthesis via inducing mitochondrial dysfunction [20]. By considering this, we hypothesized that Fumagillin may regulate mitochondrial function. Total cellular ATP, mitochondrial transcriptional activity and mitochondrial DNA content were used to evaluate mitochondrial function and energetic synthesis. As it is shown in Fig 5A, Fumagillin treatment significantly decreased ATP synthesis after 6–24 h. By considering that mitochondria is a main place that produce energy, the result indicates that Fumagillin treatment inhibits mitochondria’s energetic synthesis. Without disturbing nuclear-related transcription, Fumagillin inhibited mitochondrial transcription, including COX I, COX 3, ND1, and Cyb (Fig 5B). Furthermore, Fumagillin obviously increased JC PE-A proportion after JC-1 staining (Fig 5C). Taken together, Fumagillin decreased mitochondrial homeostasis by disturbing mitochondrial membrane potential and resulted in mitochondrial dysfunction.

RETRACTED

**Fig 5:** Fumagillin regulates mitochondrial function and homeostasis. After being treated with Fumagillin for 6–24 h, ATP synthesis (A) and mitochondrial transcriptional activity (B) were measured in Huh-7 or SNU-449 cells. *P<0.05, vs. Mock group. C. After being treated with Fumagillin for 24 h, mitochondrial homeostasis was measured by performing JC-1 staining followed by flow cytometry assay.

### Fumagillin regulates stemness of CSCs via decreasing MetAP-2

By considering that MetAP-2 is a specific target of Fumagillin [21]. Expectedly, Fumagillin treatment significantly decreased MetAP-2 transcriptionally and post-transcriptionally (Fig 6A). The expression level analyzed by GEPIA revealed MetAP-2 presents an obvious high expression in LIHC tissues compared with non-tumor tissues, and high expression level of MetAP-2 was negatively associated with overall survival rate (Fig 6B, p = 0.0081, n(low) = 218, n(high) = 146).

**Fig 6:** Fumagillin treatment decreased MetAP-2. A. After Fumagillin treatment, MetAP-2 mRNA (left panel) and protein (right panel) were measured in Huh-7 or SNU-449 CSCs. *P<0.05, vs. Mock group. B. GEPIA database presents the transcriptional level of MetAP-2 in LIHC tissues (left panel) and its relation with overall survival rate (right panel). By transfecting lentivirus, MetAP-2 was efficiently overexpressed (C, *P<0.05, vs vector group) or downregulated (D, *P<0.05, vs shScrambled group). E. Overexpressed MetAP-2 is not affected by Fumagillin treatment. F. After being treated with Fumagillin for 24 h or MetAP-2 knockdown, mitochondrial homeostasis was measured by performing JC-1 staining followed by flow cytometry assay.

To confirm whether Fumagillin affects stemness and malignant behaviors of CSCs via, at least partially, MetAP-2, we efficiently overexpressed (Fig 6C) or knockdown (Fig 6D) MetAP-2. Introduction of MetAP-2 coding sequence partially reversed Fumagillin-induced MetAP-2 decrease, indicated that post-transcriptional regulation of Fumagillin on MetAP-2 plays partial effect (Fig 6E). To further confirm whether Fumagillin regulates mitochondrial membrane potential via regulating MetAP-2, we quantitatively measured mitochondrial membrane potential after Fumagillin treatment or MetAP-2 knockdown. As presented in Fig 6F, both Fumagillin treatment and MetAP-2 knockdown increased JC-1 FITC positive proportion, indicating that Fumagillin might affect mitochondrial membrane potential via regulating MetAP-2 expression.

RETRACTED

We then further confirmed that whether Fumagillin affects stemness and malignant behaviors via downregulating MetAP-2. It is observed that, downregulation of MetAP-2 by transfecting shRNA target to MetAP2 mRNA inhibited sphere formation, expression of stemness relative markers, blocked cell cycle progression and inhibited invasion (Fig 7A–7D), which are similar with the effects of Fumagillin treatment. This indicates that Fumagillin potentially plays inhibitory roles via decrease MetAP-2. We also detected p53 and p21 expressions, which are two downstream regulated target of MetAP-2 [22,23]. As expected, Fumagillin treatment stimulated p53 activity and resulted in p21 upregulation, which is a key regulator of cell cycle blockage at G_1_/G_0_ phase. Notably, inhibition of p53 transcriptional activity induced by MetAP-2 knockdown by addition of PFT-α, a p53 transcriptional inhibitor, failed to reverse loss of mitochondrial homeostasis, demonstrating that p53 is not involved in the effect of Fumagillin on mitochondrial function (Fig 6F).

**Fig 7:** Fumagillin affects stemness, proliferation and invasion partially via downregulating MetAP-2. With the presence of Fumagillin, the effects of MetAP-2 knockdown on sphere formation (A), expression of stemness related factors (B), cell cycle distribution (C, *P<0.05, vs. shScrambled group), and cell invasion (D). After PFT-α treatment, the effects of Fumagillin on p53 and p21 was measured by performing western blot.

### 48-h treatment of Fumagillin inhibits the tumor growth of CSCs in vivo

By considering that stemness of CSCs is critical for tumorigenicity when transplanted into an animal host, CSCs were pre-treated with Fumagillin for 48 h, and same number of CSCs with Fumagillin pre-treated or untreated was injected into nude mice, respectively. As presented in Fig 8A, tumor growth was inhibited in Fumagillin-treated group compared with that of untreated group, while there was no difference in the body weight of the two groups of mice (Fig 8A, right panel). To validate the role of Fumagillin in vivo, the expression levels of MetAP-2 was confirmed, presenting that pretreatment of Fumagillin obviously decreased MetAP-2 in tumors (Fig 8B). By performing Ki67 staining, it is observed that Ki67 positive staining in Fumagillin pre-treated group was obviously decreased than that in mock group, indicating that pre-treatment inhibited proliferation of seeded tumor cells (Fig 8C). Furthermore, we also detected downstream target of MetAP2, including p53 and p21. As presented in Fig 8D, Fumagillin pre-treatment also increased P53 and P21. All these results demonstrated that Fumagillin pretreatment might decreased MetAP-2 protein level and thus upregulated P53 and P21, resulted in inhibition of tumor growth in vivo.

RETRACTED

**Fig 8:** Fumagillin pre-treatment inhibited tumor growth in nude mice. Huh-7 CSCs were pretreated with Fumagillin for 48h, then been injected into nude mice. Every five days from day 10 after injection, volume of tumors was measured (A). In tumor sections, MetAP-2 (B) and Ki67 positive staining (C) were measured by performing immunohistochemistry measured. D. MetAP-2, P53 and P21 were measured by performing western blot in tumors (n = 4 for each group). *p<0.05, vs. Mock group.

## Discussion

In this article, we showed that fumagillin exerts inhibitory effects on the formation of CSCs derived from hepatocellular carcinoma cells. This was confirmed by evaluating stemness hallmarks, including OCT4, CD44 and SOX2 expression. Moreover, fumagillin administration markedly decreased CSC malignant traits, including cell proliferation, cell cycle progression, invasion, and tumor formation. This was potentially achieved by degrading MetAP-2 without involvement of its downstream proteins p53 and p21. Furthermore, fumagillin treatment decreased the mitochondrial membrane potential, which is critical for maintaining mitochondrial homeostasis. Notably, inhibition of p53 transcriptional activity by adding PFT-α failed to reverse the inhibitory effect of fumagillin on mitochondria, indicating that fumagillin exerts antitumor effects in at least two manners. Given these results, fumagillin could be employed as a novel strategy in treating hepatocellular carcinoma by targeting a subpopulation of CSCs.

Biosynthesis studies have shown that fumagillin is produced partly by the terpene route and partly by the acetic acid route [24]. Fumagillin has been reported to act as a tumor suppressor in addition to an antibacterial effect. It strongly inhibits osteosarcoma cell lines. has been evaluated in human cancer clinical trials [25]. Together with fumaricin, these synthetic analogs target fumagillin to destroy tumor blood vessels. Although fumagillin has tumor suppressive properties, long-term use has been reported to cause side effects of weight loss [26,27]. Kin et al. [28] found that the administration of fumagillin increased liver weight relative to body weight in rats [21]. In our results, fumagillin markedly decreased the formation of spheres derived from Huh-7 and SNU-449 hepatocellular carcinoma cells. Furthermore, fumagillin exerts specific antitumor effects on CSCs by both inhibiting sphere formation and promoting the loss of stemness in CSCs. Notably, administration of fumagillin significantly inhibited tumor growth in nude mice without an obvious effect of decreasing body weight. This can be explained by the fact that instead of fumagillin administration via the intragastric route, in vitro cultured CSCs were pretreated with fumagillin for 48 h, which was then completely removed. Our results indicate that a low dose of fumagillin or other drug administration routes could be a promising strategy to avoid side effects.

RETRACTED

MetAP is a dual functional protein that plays a critical role in posttranslational processing and regulation of protein synthesis. In yeast and humans, two proteins have METAP activity, METAP1 and METAP2. MetAP2 plays an important role in the development of different types of cancer. Since MetAP2 was found to be a target molecule of the antiangiogenic compound fumagillin, more attention has been devoted to its role and mechanisms in tumorigenesis than to MetAP1. Fumagillin is considered an inhibitor of MetAP-2 by directly inducing degradation. Moreover, by employing the GEPIA online analysis tool, it is presented that relatively higher expression of MetAP-2 is positively correlated with poor overall survival and disease-free survival rates, indicating that fumagillin might exert anti-CSC effects via, at least partially, downregulating MetAP-2. As expected, the degradation of MetAP-2 induced by fumagillin was reversed by transfection with the MetAP-2 coding plasmid, indicating that MetAP-2 is posttranscriptionally regulated by fumagillin. Regulation of MetAP-2 by fumagillin is potentially a main cause of mitochondrial dysfunction. However, it is still a limitation that we failed to point out whether the regulation of stemness by fumagillin occurs by regulating MetAP-2, which is worth investigating in further analysis.

We proposed new antitumor effects of fumagillin by targeting stem-like cells in hepatocellular carcinoma and subsequently inhibiting stemness. Downregulating the expression of stemness hallmark genes, including OCT4, CD44 and SOX2, denoted malignant differentiation in producing mature cancer cells. In addition, we also showed the effects of fumagillin on mitochondrial homeostasis by decreasing the mitochondrial membrane potential without elucidating the exact mechanism. This study may offer a novel treatment strategy for cancer by targeting CSCs, hence having important scientific significance and potential clinical application value.

RETRACTED

## Supporting information

S1 Raw images (PDF)
